This article has been retracted.

# Inhibitors of apoptosis proteins in experimental benign prostatic hyperplasia: effects of serenoa repens, selenium and lycopene

**DOI:** 10.1186/1423-0127-21-19

**Published:** 2014-03-10

**Authors:** Letteria Minutoli, Domenica Altavilla, Herbert Marini, Mariagrazia Rinaldi, Natasha Irrera, Gabriele Pizzino, Alessandra Bitto, Salvatore Arena, Sebastiano Cimino, Francesco Squadrito, Giorgio Ivan Russo, Giuseppe Morgia

**Affiliations:** 1 Department of Clinical and Experimental Medicine, University of Messina, Messina 98125, Italy; 2 Department of Paediatric, Gynaecological, Microbiological and Biomedical Sciences, University of Messina, Messina 98125, Italy; 3 Department of Urology, Polyclinic Hospital, University of Catania, Catania 95100, Italy

**Keywords:** Apoptosis, BPH, IAPs, Lycopene, Selenium, *Serenoa Repens*

## Abstract

**Background:**

The apoptosis machinery is a promising target against benign prostatic hyperplasia (BPH). Inhibitors of apoptosis proteins (IAPs) modulate apoptosis by direct inhibition of caspases. *Serenoa Repens* (SeR) may be combined with other natural compounds such as Lycopene (Ly) and Selenium (Se) to maximize its therapeutic activity in BPH. We investigated the effects of SeR, Se and Ly, alone or in association, on the expression of four IAPs, cIAP-1, cIAP-2, NAIP and survivin in rats with experimental testosterone-dependent BPH. Moreover, caspase-3, interleukin-6 (IL-6) and prostate specific membrane antigen (PSMA) have been evaluated.

Rats were administered, daily, with testosterone propionate (3 mg/kg/sc) or its vehicle for 14 days. Testosterone injected animals (BPH) were randomized to receive vehicle, SeR (25 mg/kg/sc), Se (3 mg/kg/sc), Ly (1 mg/kg/sc) or the SeR-Se-Ly association for 14 days. Animals were sacrificed and prostate removed for analysis.

**Results:**

BPH animals treated with vehicle showed unchanged expression of cIAP-1 and cIAP-2 and increased expression of NAIP, survivin, caspase-3, IL-6 and PSMA levels when compared with sham animals. Immunofluorescence studies confirmed the enhanced expression of NAIP and survivin with a characteristic pattern of cellular localization. SeR-Se-Ly association showed the highest efficacy in reawakening apoptosis; additionally, this therapeutic cocktail significantly reduced IL-6 and PSMA levels. The administration of SeR, Se and Ly significantly blunted prostate overweight and growth; moreover, the SeR-Se-Ly association was most effective in reducing prostate enlargement and growth by 43.3% in treated animals.

**Conclusions:**

The results indicate that IAPs may represent interesting targets for drug therapy of BPH.

## Background

Apoptosis plays an important role in the control of cell growth and in the maintenance of tissue homeostasis [1]. Programmed cell death comprises a series of molecular steps that culminate in the clearance of impaired and altered cells, avoiding at the same time the leaking of deleterious substances into the surrounding tissues [2,3].

Benign prostatic hyperplasia (BPH) is a common cause of bothersome lower urinary tract symptoms (LUTS). The burden of BPH on healthcare systems and to society is already high and it is expected to increase in line with the greater life expectancy [4,5]. BPH results from smooth muscle and epithelial proliferation primarily within the prostatic transition zone that can produce LUTS [6-9]. As a consequence, targeting apoptosis may represent a rational therapeutic strategy in the treatment of BPH.

Emerging contributors in this context are the inhibitors of apoptosis proteins (IAPs), which halt cell death in response to diverse stimuli [10]. IAPs influence apoptosis by direct inhibition of caspases and modulation of the transcription factor Nuclear Factor-κB (NF-κB). Eight mammalian IAPs are known at present: X-chromosome-linked IAP (XIAP), cellular IAP-1 and IAP-2 (cIAP-1 and cIAP-2), neuronal apoptosis inhibitory protein (NAIP), survivin, BRUCE, livin and testis-specific IAP (Ts-IAP). Increased IAPs expression has been shown in pathological human prostate including benign hyperplasia, prostatic intraepithelial neoplasia and cancer [11].

Phytotherapeutic supplements, mainly based on Saw Palmetto-derived *Serenoa Repens* (SeR), are numerous and used frequently; however, data supporting efficacy are limited, making treatment recommendations difficult [12]. SeR is often associated with other natural compounds such as Lycopene (Ly), a carotenoid, and Selenium (Se), an essential trace element, to maximize its therapeutic activity in BPH [13].

Previous data have shown that triple SeR-Se-Ly combination is more effective than therapy with SeR alone in reawakening apoptosis and in dumping hormone-dependent prostatic growth [14]. In order to better understand the molecular mechanism(s) of the triple therapeutic association SeR-Se-Ly on apoptosis, we studied the effects of SeR, Se and Ly, alone or in association, on the expression of four IAPs, cIAP-1, cIAP-2, NAIP and survivin in rats with experimental testosterone-dependent BPH. Moreover, caspase-3, interleukin-6 (IL-6) and prostate specific membrane antigen (PSMA) have been also evaluated.

## Methods

### Ethics statement

All procedures complied with the standards for care and use of animal subjects as stated in the Guide for the Care and Use of Laboratory Animals and the protocol was reviewed and approved by the Ethics Committee of the University of Messina. All efforts were made to minimize animals suffering.

### Animals

Male Sprague-Dawley rats aged 3 months and weighing 220-250 grams were purchased from Charles River Laboratories, Italy. After 1 week of stabilization, animals were randomly assigned to 6 groups: Sham administered with vehicle (100 μl corn oil subcutaneously), BPH receiving testosterone propionate (3 mg/kg/sc diluted in corn oil in a volume of 100 μl), BPH + SeR injected with SeR (25 mg/kg/sc in corn oil), BPH + Ly injected with Ly (1 mg/kg/sc, in corn oil), BPH + Se injected with Se (3 mg/kg/sc, in corn oil) and BPH + Ly-Se-SeR administered with the combination of Ly-Se-SeR for 14 days [14,15]. Each treatment group included seven animals. At the end of the experiment, animals were sacrificed under ether anaesthesia and their prostates immediately removed for further analysis.

### Prostate weight

After removal, prostates were weighed and percentage of growth inhibition was calculated as follows: 100− [(TG (treated group) − Sham)/(BPH − Sham) × 100], where TG were the values of the treated groups.

### Isolation of cytoplasmic proteins and determination of IAPs and caspase-3

Isolation and determination of cytoplasmic proteins were performed as previously described [16]. The concentration of total proteins was determined using a Bio-Rad® protein assay kit. cIAP-1, cIAP-2, survivin (Cell Signaling), NAIP and caspase-3 (Abcam) expression were evaluated by Western Blot. The IAPs and caspase-3 protein signal was quantified by scanning densitometry using a bioimage analysis system (Bio-Profil).

### Histology

Prostates were routinely processed and embedded in paraffin, and 5 μm-thick sections were cut and stained with haematoxylin-eosin [14,16].

### Immunofluorescence

Samples were fixed in 4% paraformaldehyde, dehydrated, embedded and sectioned at 5 μm. The sections were pre-incubated with 1% bovine serum albumin (BSA), 0.3% Triton X-100 in PBS, for 15 min, at room temperature. In order to evidence smooth muscle cells, double-localization reactions were performed incubating, in the same section, goat anti-smooth muscle alpha-actin antibody (GeneTex, Inc, diluted 0.1-0.3 μg/ml) with rabbit survivin or NAIP antibodies, respectively. After washing with PBS, the sections were incubate with Alexa Fluor 488 (for anti-smooth muscle alpha-actin) or 594 (for survivin or NAIP) secondary antibodies. 4′,6-diamidino-2-phenylindole (DAPI) (Sigma Chemicals) was used for nuclear staining diluted 1:1000 in PBS for 10 min. Finally, slides were washed in PBS and sealed with mounting medium. The sections were then analysed and images acquired using a confocal microscopy.

### Immunohistochemistry

At the scheduled time point, animals were sacrificed and specimens of prostatic tissue were excised and left in 10% buffered formalin for at least 24 hrs before ascending the alcohol grade and being included in paraffin at 60-65°C. Slices of 5 μm were rehydrated in graded alcohol, antigen retrieval was performed with pH 6.0 buffer citrate and endogenous peroxidase (i.e. from red blood cells) blocking with 1% H_2_O_2_ in PBS. Primary antibody (PSMA and caspase-3, Cell Signaling) was incubated overnight at 4°C in a moisturized chamber and the day after secondary antibody (Pierce anti-rabbit) was added and reaction visualized with 3,3′-Diaminobenzidine (DAB) (Sigma-Aldrich, Milan, Italy). Counterstaining was performed in Haematoxylin DAB. Negative control slices were tested using PBS instead of primary antibody. The samples were coded and the operator was blinded during the analysis.

### Real-Time PCR (qRT-PCR)

For the gene expression study, the extraction of total mRNA was performed from tissue prostate using TRIZOL (Invitrogen, Milan, Italy) under sterile conditions, following the manufacturer’s protocol. For each sample, 5 μg of mRNA were reverse transcripted into cDNA and 3 μl of cDNA were amplified in duplicate with the TaqMan Universal PCR Master Mix containing primer and specific probes (TaqMan), then using the instrument SDS 7300 Real Time PCR (Applied Biosystems, Foster City, CA). The reversed transcribed product was used to quantify the amount of IL-6. The result was expressed as number of copies of the target gene compared to the housekeeping gene (β-actin).

### Statistical analysis

Comparison between groups was performed using the Kruskal-Wallis one-way test. Differences between individual treatment groups were compared using Dunn’s test. P <0.05 was considered significant. Statistical analysis were performed using GraphPad Prism software version 5.0 for Windows.

## Results

### cIAP- 1, cIAP-2, NAIP, Survivin and caspase-3 expression by Western Blot

BPH animals treated with either vehicle or other compounds showed unchanged expression of cIAP-1 and cIAP-2 compared to sham animals (data not shown). NAIP and survivin were significantly augmented in prostate tissues from vehicle treated BPH animals when compared with sham animals and the treatment with SeR, Se or Ly markedly reduced their expression. However, the effect of Ly was greater than those of either SeR or Se. Furthermore, SeR-Se-Ly combination was the most effective in reducing NAIP and survivin expression (Top panel, Figure 1A and B). Caspase-3 was more expressed in BPH prostates than in sham prostates. Ly produced a greater increase of caspase-3 than SeR and Se while SeR-Se-Ly association caused the highest induction (Top panel, Figure 1C).

**Figure 1:** **Expression of IAPs, NAIP, Survivin and caspase-3 in the Western Blot and Immunohistocehemical analysis.***Top Panel:* Representative Western Blot analysis of NAIP **(A)**, survivin **(B)** and caspase-3 **(C)**. The prostate is collected from Sham rats treated with vehicle and BPH rats treated with either vehicle or SeR (25 mg/Kg) or Se (3 mg/kg) or Ly (1 mg/kg) or Ser + Se + Ly *p < 0.01 vs Sham; #p < 0.05 vs BPH + vehicle; •p < 0.01 vs BPH + vehicle; §p < 0.001 vs BPH + vehicle. Bars represent the mean ± SEM of seven experiments. ***Bottom Panel: *Immunhistochemical detection of Caspase-3.** The prostate is collected from Sham rats treated with vehicle **(D)** and BPH rats treated with either vehicle **(E)** or SeR (25 mg/Kg) **(F)** or Se (3 mg/kg) **(G)** or Ly (1 mg/kg) **(H)** or SeR + Se + Ly **(I)**. Immunohistochemistry for caspase-3 showed a negative reaction in sham **(D)**. In BPH rats treated with vehicle **(E)**, a focal cytoplasmatic positivity was documented in acini and stromal cells. A progressive enhancement of positivity was observed in BPH rats treated with SeR **(F)**, Se **(G)**, Ly and with the combination of SeR + Se + Ly **(I)**, where it reached the highest expression. Original magnification ×400.

### Caspase-3 detection by immunohistochemical analysis

Immunohistochemistry for caspase-3 showed a negative reaction in sham animals (Bottom Panel, Figure 1D). while prostate samples of BPH rats treated with vehicle showed a focal cytoplasmatic positivity in acini and stromal cells (Bottom Panel, Figure 1E). The treatment with SeR, Se or Ly in BPH rats markedly augmented the positivity for Caspase-3 (Bottom Panel, Figure 1F-H). However, the SeR-Se-Ly combination was the most effective in increasing prostate Caspase-3 expression (Bottom Panel, Figure 1I).

### Histology

We showed a full derangement of the prostate tissue and a profound hyperplasia in BPH vehicle-treated animals compared with sham animals. SeR, Se and Ly decreased the impaired histological pattern and the marked hyperplasia. The Ly showed a better protection than SeR and Se and the SeR-Se-Ly combination was most effective in reducing prostate hyperplasia (Figure 2).

**Figure 2:** **Histological findings.** Sham prostate treated with vehicle showing regular acini with cubodail epithelium with round nuclei showing a regular alignment **(A)**. BPH prostate treated with vehicle showed irregular acinar shape with villous projection into the lumen and foci of piling-up hyperplastic nodule with loss of epithelial polarity are evident. The epithelium is cylindric/cuboidal and round/ovoid nuclei are irregularly aligned. Presence of hard stroma and an intact basal layer surrounding the acini **(B)**. Similarly, BPH prostate treated with SeR and Se displayed cilindric/cuboidal epithelial cells but villous projections are just slightly present or absent, respectively. Moderate stroma and intact basal layer around the acini **(C-D)**. Treatment with Ly proved cuboidal epithelial cells, absence of villous projection and the presence of moderate stroma with intact basal layer around the acini **(E)**. Differently, BPH prostate treated with the combination SeR-Se-Ly resembled the histological features of a normal acinar structure **(F)** (Original magnification ×100 and ×400 in the box).

### Immunofluorescence analysis

We documented a diffuse and marked membrane and cytoplasmatic expression of NAIP in prostatic epithelium of BPH when compared with sham rats (Figure 3A-a and B-a). Several treatments decreased NAIP expression, but Ly showed a greater effect than SeR and Se while the SeR-Se-Ly association produced the highest inhibition (Figure 3C-a, D-a, E-a and F-a).

**Figure 3:** **Immunofluorescence analysis of NAIP and Survivin.** Immunofluorescence stainings of NAIP **(a)** and Survivin **(b)** (in red) and anti-smooth muscle alpha-actin (in green) showed a diffuse positivity in BPH prostatic epithelium treated with vehicle **(B)**. In a lesser extent, the fluorescence was present in BPH prostate treated with SeR, Se and Ly, in a decremental fashion **(C, D** and **E)**. Differently, NAIP and Survivin were just focally or not detected in Sham and BPH prostate treated with the combination SeR-Se-Ly **(A** and **F, respectively)** (Original magnification ×400).

We found that survivin was localized inside the cytoplasm, as diffuse spots, and likely in the mitochondria. The fluorescence was markedly augmented in vehicle-treated BPH specimens than in prostate tissues from sham animals (Figure 3A-b and B-b). SeR, Se and Ly reduced NAIP expression, being Ly the most effective among the isolated treatments (Figure 3C-b, D-b and E-b). The SeR-Se-Ly association induced the greatest inhibition on survivin fluorescence (Figure 3F-b).

### Prostate growth

Table 1 shows that prostate weight augmented at the end of testosterone administration. The administration of SeR, Se and Ly significantly blunted prostate overweight and growth and the SeR-Se-Ly association was the most effective in reducing growth by 43.3% in treated animals.

**Table 1:** Effects of treatments on prostate growth in rats treated with testosterone

**Group**	**Prostate weight (grams)**	**Growth inhibition (%)**
Sham	0.81 ± 0.06	-
BPH + vehicle	1.55 ± 0.03	-
BPH + SeR	1.02 ± 0.07*	34.2%*
BPH + Se	1.01 ± 0.08*	34.9%*
BPH + Ly	0.98 ± 0.05*	36.8%*
BPH + Ly-Se-SeR	0.88 ± 0.04^#^	43.3%^#^

*p < 0.005 vs BPH + vehicle; #p < 0.001 vs BPH + vehicle.

### Prostatic IL-6 mRNA expression

Prostates from sham animals treated with vehicle had basal levels of IL-6 evaluated as mRNA expression (Top panel, Figure 4). Prostate tissue from BPH rats showed a significantly increase in IL-6 mRNA compared to sham animals. The treatment with SeR, Se or Ly markedly reduced prostate IL-6 mRNA expression. However, the effect of Ly was greater than those of either SeR or Se. Furthermore, SeR-Se-Ly combination was the most effective in reducing prostate IL-6 expression (Top panel, Figure 4).

**Figure 4:** **IL-6 mRNA expression and Immunohistochemical analysis of PSMA.***Top Panel:* Expression of mRNA for IL-6. The prostate is collected from Sham rats treated with vehicle and BPH rats treated with either vehicle or SeR (25 mg/Kg) or Se (3 mg/kg) or Ly (1 mg/kg) or Ser + Se + Ly *p < 0.01 vs Sham; #p < 0.05 vs BPH + vehicle; •p < 0.01 vs BPH + vehicle; §p < 0.001 vs BPH + vehicle. Bars represent the mean ± SEM of seven experiments. ***Bottom panel: *Immunohistochemical detection of PSMA.** The prostate is collected from Sham rats treated with vehicle **(A)** and BPH rats treated with either vehicle **(B)** or SeR (25 mg/Kg) **(C)** or Se (3 mg/kg) **(D)** or Ly (1 mg/kg) **(E)** or SeR + Se + Ly **(F)**. Immunohistochemistry for PSMA showed a negative reaction in sham **(A)** as well as in BPH treated with Ly **(E)** or with the combination SeR + Se + Ly **(F)**. Differently, a moderate cytoplasmatic positivity was observed in acini and stromal cells of BPH rats treated with vehicle **(B)** and, in a lesser extent, of BPH rats treated with SeR **(C)** or Se **(D)**. Original magnification ×400.

### Immunohistochemical analysis of PSMA

Immunohistochemistry for PSMA showed a negative reaction in sham animals ( Bottom panel, Figure 4A) as well as in BPH rats treated with Ly (Bottom panel, Figure 4E) or with the combination SeR-Se-Ly (Bottom panel, Figure 4F). By contrary, prostate samples of BPH rats treated with vehicle showed a moderate cytoplasmatic positivity (Bottom panel, Figure 4B). Similar picture, although to a lesser extent, was revealed in BPH rats treated with SeR or Se (Bottom panel, Figure 4C and D).

## Discussion

Disturbances in apoptosis have been linked to number of human medical diseases and conditions, including BPH. SeR is the most frequently used phyto-therapeutic agent in the treatment of BPH. Besides SeR, Ly has been shown to improve prostate health and its anti-proliferative effects in BPH seems to be due to an increased number of apoptotic cells. It has been suggested that the lipido-sterolic extract of this natural agent increases bax/bcl-2 ratio and caspase-3 activity in prostatic specimens from BPH patients [17]. This effect has been confirmed in both hormone-sensitive or hormone-insensitive human carcinoma cells [18,19]. Furthermore, it has been shown that SeR-Se-Ly association is superior to SeR alone for decreasing hormone-dependent prostatic growth and it is likely that this greater effect might derive from a more robust induction of programmed cell death.

Manipulating poor apoptosis could represent a rational strategy for the management of BPH. To this regard, IAPs family plays a key role in apoptosis through their ability to inhibit caspases [20]. As far as we know, there is no study that investigated so far IAPs in BPH after treatment with SeR, Se and Ly, alone or in association. The cIAP-1 and cIAP-2 were originally identified through their ability to bind to tumour necrosis factor-associated factor 2 (TRAF2) [21]. Though TRAF2 interactions, cIAP-1 and cIAP-2 are recruited to TNFRI and TNFRII associated complexes where they regulate apoptosis [22]. Therefore, cIAP-1 and cIAP-2 are mainly involved in the regulation of the extrinsic pathway of the apoptosis, through the blockade of caspase-8 activation. BPH animals did not display a significant increased expression of cIAP-1 and cIAP-2 when compared with sham animals, thus suggesting that these two IAPs are not involved in the apoptosis disturbance in the benign overgrowth of the prostate gland. In addition SeR, Se and Ly, either alone or in association, did not modify cIAP-1 and cIAP-2 expression. These findings also led us to hypothesize that in BPH the impairment in the extrinsic pathway does not seem to contribute to the disturbed cell death program.

NAIP was identified in 1995 and it impairs apoptosis by inhibition of the executioner caspases-3 and -7 [23,24]. Interestingly, human normal prostates do not express measurable basal levels of NAIP; by contrast, enhanced expression of NAIP has been shown in human BPH and prostate cancer [11]. Therefore, NAIP is an IAP that appears to be selectively enhanced in the benign and malign overgrowth of the prostate, thus unmasking for it a key role in the dumping of the apoptosis that occurs in these two pathological conditions. In agreement with these findings, we found an increased expression of NAIP in the prostates harvested from vehicle-treated BPH animals. SeR, Se and Ly, either alone or in association, significantly reduced NAIP expression. Ly caused a greater inhibition than SeR and Se and the SeR-Se-Ly caused the highest inhibition of NAIP. We also investigated the executioner caspase-3 by western blot analysis and, through immunohistochemical analysis, we confirmed that inhibition of NAIP paralleled an enhanced expression of pro-apoptotic protein.

Survivin has a central role in the negative regulation of apoptosis, however the exact mechanism by which survivin dumps programmed cell death is still far from being fully understood [25]. Indeed, survivin has been shown to inhibit the executioner caspase-3 [26]. In our model of prostate enlargement induced by testosterone we found an enhanced expression of survivin. This latter is in agreement with previous findings in humans [11]. The administration of SeR, Se and Ly, either alone or in association, significantly blunted survivin expression. As observed for NAIP, Ly caused a more profound reduction of survin expression than SeR and Se; furthermore the SeR-Se-Ly association produced the greatest inhibition of survivin expression. Altogether, these findings point out the key role played by survivin in the negative regulation of apoptosis during prostate growth following testosterone administration, confirming that this IAP might represent an interesting target for drug therapy.

Moreover, inflammation plays a crucial role in BPH. Recent insights into the pathogenesis of BPH highlighted the differential expression of cytokines in BPH tissue suggesting a role for inflammation in the propagation of BPH [27]. Additionally, Rick *et al*. have demonstrated that a luteinizing hormone-releasing hormone antagonist inhibits the gene expression of proinflammatory cytokines in a rat model of BPH [28].

As a matter of fact, our data revealed an increased expression of IL-6 levels in prostate samples harvested by vehicle-treated BPH when compared with sham animals. By contrary, the therapeutic combination of SeR-Se-Ly significantly reduced IL-6 levels, then confirming the anti-inflammatory role of therapeutic cocktail.

The combined treatment with SeR-Se-Ly was more effective than the single treatments in preventing the histological features of BPH and inhibiting growth by 43.3%, suggesting that Se and Ly, at pharmacological doses, further enhances SeR efficacy in BPH. Our data show that the enhancing efficacy of the association may be a direct consequence of a more pronounced ability of the association in reawakening the apoptosis program, as also supported by reduced levels of PSMA in animals treated with SeR-Se-Ly, and identify in the inhibition of NAIP and survivin the molecular mechanism by which this task is accomplished. Interestingly, immunofluorescence experiments show that expression of NAIP is evident in the cytoplasm of prostatic cell epithelium while survivin is localized inside the cytoplasm and in the mitochondria.

Overall, among the three compounds, Ly appears to give the major contribution in maximizing the effects of SeR-Se-Ly; in fact, it caused the higher inhibitory effect on IAPs than Se and SeR, alone.

## Conclusions

Benign prostatic hyperplasia (BPH) is a common cause of bothersome LUTS in men, representing a growing entity in terms of healthcare costs and morbidity.

Despite medical therapy improves LUTS plant extracts have been used in the medical management of this medical condition with the aim to relieve symptoms without adverse events related to treatment.

In the current study, we demonstrated that the combined treatment with SeR-Se-Ly was more effective than the single treatments in preventing the histological features of BPH suggesting that Se and Ly, at pharmacological doses, further enhances SeR efficacy in BPH. The inhibition of the apoptosis in BPH could be a targeted therapy to relief patients from LUTS, although more research in humans is needed to confirm these findings.

## Abbreviations

BPH: Benign prostatic hyperplasia; cIAP-1 and cIAP-2: Cellular IAP-1 and IAP-2; IAPs: Inhibitor of apoptosis proteins; IL-6: Interleukin-6; Ly: Lycopene; LUTS: Lower urinary tract symptoms; NAIP: Neuronal apoptosis inhibitory protein; NF-κB: Nuclear Factor-κB; PSMA: Prostate specific membrane antigen; Se: Selenium; SeR: *Serenoa Repens*; TRAF2: Necrosis factor-associated factor 2; Ts-IAP: Testis-specific IAP; XIAP: Chromosome-linked IAP.

## Competing interests

The authors do not have any conflict of interests.

## Authors’ contributions

LM, DA, HM, FS, & GM designed the research study; LM, HM & FS wrote the paper; MR, NI, GP & SA analyzed and interpreted the data; AB, SC & GIR contributed to critical revision of the article; LM, FS & GM obtained and provided administrative, technical or logistic support. All authors approved the manuscript.
